The article "Parathyroid hormone promotes the osteogenesis of lipopolysaccharide-induced human bone marrow mesenchymal stem cells through the JNK MAPK pathway" was published in 2021. Journal: Biosci Rep.

# Parathyroid hormone promotes the osteogenesis of lipopolysaccharide-induced human bone marrow mesenchymal stem cells through the JNK MAPK pathway

**DOI:** 10.1042/BSR20210420

**Published:** 2021-08-20

**Authors:** Ziyue Qin, Shu Hua, Huifen Chen, Zhuo Wang, Haoran Wang, Jiamin Xu, Yuli Wang, Wu Chen, Weina Zhou

**Affiliations:** 1 Department of Periodontology, The Affiliated Stomatological Hospital of Nanjing Medical University, Nanjing, China; 2 Jiangsu Province Key Laboratory of Oral Diseases, Nanjing Medical University, Nanjing, China; 3 Jiangsu Province Engineering Research Center of Stomatological Translational Medicine, Nanjing, China; 4 Department of Temporomandibular Joint, The Affiliated Stomatological Hospital of Nanjing Medical University, Nanjing, China; 5 Department of Endodontics, The Affiliated Stomatological Hospital of Nanjing Medical University, Nanjing, China; 6 Department of Oral and Maxillofacial Surgery, The Affiliated Stomatological Hospital of Nanjing Medical University, Nanjing, China

**Keywords:** Human bone marrow mesenchymal stem cells, Lipopolysaccharides, Mitogen-activated protein kinase signaling pathway, Osteogenic differentiation, Parathyroid hormone

## Abstract

Periodontitis is a series of inflammatory processes caused by bacterial infection. Parathyroid hormone (PTH) plays a critical role in bone remodeling. The present study aimed to investigate the influences of PTH on human bone marrow mesenchymal stem cells (HBMSCs) pretreated with lipopolysaccharide (LPS). The proliferative ability was measured using cell counting kit-8 (CCK-8) and flow cytometry. The optimal concentrations of PTH and LPS were determined using alkaline phosphatase (ALP) activity assay, ALP staining, and Alizarin Red staining. Osteogenic differentiation was further assessed by quantitative reverse-transcription polymerase chain reaction (RT-qPCR), Western blot analysis, and immunofluorescence staining. PTH had no effects on the proliferation of HBMSCs. Also, 100 ng/ml LPS significantly inhibited HBMSC osteogenesis, while 10^−9^ mol/l PTH was considered as the optimal concentration to reverse the adverse effects. Mechanistically, c-Jun N-terminal kinase (JNK) phosphorylation was activated by PTH in LPS-induced HBMSCs. SP600125, a selective inhibitor targeting JNK mitogen-activated protein kinase (MAPK) signaling, weakened the effects of PTH. Taken together, the findings revealed the role and mechanism of PTH and JNK pathway in promoting the osteogenic differentiation of LPS-induced HBMSCs, which offered an alternative for treating periodontal diseases.

## Introduction

Periodontitis is a group of chronic inflammatory processes characterized by uncoordinated immune-inflammatory reactions, which has become a common cause of tooth loss in adults [1]. So far, no effective strategies have been developed to treat periodontitis. Lipopolysaccharide (LPS), a cell wall component of Gram-negative bacteria, presents as a major nexus for virulence in the pathogenesis of periodontitis [2,3]. Human bone marrow mesenchymal stem cells (HBMSCs) obtained from human bone marrow play a key role in cell-based therapies due to their remarkable functional nature [4,5]. HBMSCs can maintain low anti-inflammatory properties under the undifferentiated state and exhibit better bone formation capability during osteoblastic differentiation [6–8]. However, the LPS-induced local inflammatory environment increases the secretion of inflammatory factors and up-regulates the oxidative stress level [9,10], leading to an inadequate biologic behavior of HBMSCs during differentiation. Therefore, discovering desirable strategies to promote HBMSC osteogenesis against an inflammatory environment is urgently needed.

Parathyroid hormone (PTH), an endocrine factor secreted by the parathyroid gland, has significant effects in terms of regulating bone metabolism and has been used as the only approved therapy by the Food and Drug Administration for osteoporosis in the United States [11]. The secretion and synthesis of PTH are sensitively controlled by the calcium concentration detection mechanism. PTH exerts anabolic effects on both osteoblasts and osteocytes by regulating bone remodeling [12]. A previous study reported that PTH guided osteoblast lineage by influencing phenotypes through reducing cell apoptosis and increasing cell viability and differentiation potential [13]. Recent studies established that the intermittent delivery of PTH led to the up-regulated osteoblast activity and down-regulated osteoblast apoptosis in the bone marrow [14–16]. Nevertheless, the effects and the underlying mechanisms of PTH responsible for remolding LPS-inhibited osteogenesis have not been fully elucidated yet. The activation of mitogen-activated protein kinase (MAPK) signals are involved in multiple physiological processes, including cell cycle control, apoptosis, and cell fate specification [17,18]. Moreover, MAPKs are often activated under inflammatory conditions, such as substances containing LPS [19]. Therefore, the present study was performed to investigate the role of PTH on the MAPK signaling pathway in LPS-induced HBMSCs.

The present study aimed to uncover the regulatory effects of PTH in the osteogenic differentiation of HBMSCs under inflammatory conditions. The role of c-Jun N-terminal kinase (JNK) MAPK was also evaluated. This might lay a foundation for the therapy of chronic inflammatory processes and expand the understanding of the impact of PTH on bone regeneration.

## Materials and methods

### HBMSC isolation, LPS treatment, and PTH administration

The present study was approved by the ethics committee of the Affiliated Hospital of Stomatology, Nanjing Medical University. The mandible samples of 80 patients, aged 20–30 years, treated by sagittal split ramus osteotomy (SSRO) in the Oral and Maxillofacial Surgery of the Affiliated Hospital of Stomatology, Nanjing Medical University were harvested. HBMSCs were isolated and cultured routinely, as reported in a previous study [20]. The isolated HBMSCs were maintained in Dulbecco’s modified Eagle’s medium (DMEM) (HyClone, U.S.A.) containing 10% fetal bovine serum (FBS; Gibco, Life Technologies), 100 U/l penicillin, and 100 µg/l streptomycin (Gibco). The cell culture was conducted in a humid environment with 5% CO_2_ at 37°C. The medium was refreshed every 2 days, and the cells from three to six passages were used for the following experiments. HBMSCs (5 × 10^4^ cells) were seeded on six-well culture plates (Corning). When the cell attachment reached 80%, HBMSCs were subjected to a 24-h treatment with serum-free medium or LPS (1 μg/ml) as previously described [21]. After 24 h, HBMSCs were washed with phosphate-buffered saline (PBS) and exposed to human PTH (1–34) (ApexBio, A1129). SP600125, a highly selective inhibitor of JNK signaling, was prepared in DMSO and used in the signaling inhibition assay. To eliminate the influence of SP600125 on PTH, LPS-induced HBMSCs were treated with SP600125 for 24 h after incubating in LPS before PTH treatment. All study protocols were approved by the ethics and research Committee of Nanjing Medical University. The permit number of the ethics committee is PJ2019-059-001. Informed consents were obtained from each participant.

### Cell proliferation assay

The cell proliferation was assessed using cell counting kit-8 (CCK-8) and flow cytometry. At the appointed time points, HBMSCs and HBMSCs treated with LPS or LPS + PTH were incubated with CCK-8 reagent (Dojindo, Kyushu Island, Japan) at 37°C for 2 h. The optical density (OD) was detected using a microplate reader (Bio-Tek, VT, U.S.A.) based on absorbance at 405 nm. Then, the cell cycle distribution (G_0_, G_1_, S, and G_2_ M phases) was evaluated using an FACScan flow cytometer (BD Biosciences, U.S.A.) and quantitated using MODFIT LT 3.2 (Verity Software House, U.S.A.).

### Alkaline phosphatase activity assay and alkaline phosphatase staining

Osteogenic differentiation was induced in osteogenic media containing 100 nM dexamethasone, 10 mM β-glycerophosphate, and 100 nM ascorbic acid (Sigma Chemical Co., U.S.A.) for 7 days. Alkaline phosphatase (ALP) activity was detected using an ALP activity kit (Nanjing Jiancheng, Nanjing, China) based on the absorbance at 405 nm as previously reported [22]. Total protein was quantitated with a BCA kit (Beyotime, Shanghai, China), and the enzymatic activity was normalized by total cellular protein concentrations among the samples. For ALP staining, HBMSCs were fixed with 70% ethanol and stained using a BCIP/NBT ALP color development kit (Beyotime). The images were photographed under phase-contrast microscopy (Epson printer, Japan).

### Alizarin Red staining

Osteogenic differentiation was induced for 14 days. The cells were fixed with 70% ethanol and stained with 2% Alizarin Red (pH = 4.2; Sigma, U.K.). The images were captured under a microscope (Epson printer).

### Quantitative real-time reverse-transcription polymerase chain reaction

The cellular RNA was extracted from cells using TRIzol reagent (Invitrogen, U.S.A.) and reverse transcribed using a reverse transcription kit (Applied Biosystems, CA, U.S.A.). Next, qRT-PCR was performed with SYBR Green Master Mix (Roche, Switzerland) on an ABI Prism 7500 real-time PCR system (Applied Biosystems) at 95°C for 30 s, followed by 40 cycles at 95°C for 5 s and 60°C for 31 s [23]. Table 1 summarizes the cDNA sequences, and GAPDH was employed as an internal reference. Data analysis was carried out by the 2^−ΔΔ*C*_t_^ method.

**Table 1:** Primers employed for quantitative real-time reverse-transcription polymerase chain reaction

Gene	Forward primer (5′–3′)	Reverse primer (5′–3′)
*ALP*	AGAACCCAAAGGCTTCTTC	CTTGGCTTTTCCTTCATGGT
*COL1*	GGACACAATGGATTGCAAGG	TAACCACTGCTCCACTCTGG
*OPN*	CAGTTGTCCCCACAGTAGACAC	GTGATGTCCTCGTCTGTAGCATC
*OCN*	AGCAAAGGTGCAGCCTTTGT	GCGCCTGGGTCTCTTCACT
*RUNX2*	TCTTAGAACAAATTCTGCCCTTT	TGCTTTGGTCTTGAAATCACA
*GAPDH*	GAAGGTGAAGGTCGGAGTC	GAGATGGTGATGGGATTTC

### Western blot analysis

Western blot analysis was carried out as previously reported [24]. Primary antibodies used were as follows: anti-runt-related transcription factor 2 (RUNX2) (#12556), ERK1/2 (#4695), anti-p-ERK1/2 (#4370), anti-JNK (#9252), anti-p-JNK (#9255), anti-p38 (#8690), anti-p-p38 (#4511), and anti-β-actin (#3700) (Cell Signaling Technology, U.S.A.), anti-ALP (ab83259), anti-osteocalcin (OCN) (ab133612) (1:1000), anti-collagen 1 (COL1) (ab34710), and anti-osteopontin (OPN) (ab8448) (Abcam, U.K.) primary antibodies. β-actin served as an internal control. The relative densitometry analysis of the phosphorylation level was carried out using ImageJ software. The relative protein level was quantified as the ratio of the level of the target protein to the level of β-actin, in each group.

### Immunofluorescence

Immunofluorescence staining was carried out as previously reported [25]. After incubation with the primary antibodies [anti-OCN (1:200) and anti-Runx2 (1:500); Abcam, U.K.] at 4°C overnight, the cells were incubated with the following secondary antibody for 1 h: Alexa Fluor 594 (1/1000; Abcam, U.K.). The nuclei were counterstained with DAPI solution (Invitrogen). The images were visualized under an inverted fluorescence microscope (Olympus, Shanghai, China).

### Statistical analysis

The experiments were all carried out for at least three times. Representative data were displayed as mean ± standard deviation (SD). SPSS 20.0 software (SPSS Inc., U.S.A.) was employed for data analysis. Differences between two groups were evaluated by the two-tailed Student’s *t* test. ANOVA was used to determine significance between multiple groups. A *P*-value <0.05 indicated a statistically significant difference.

## Results

### Effects of LPS on the growth and osteogenic differentiation of HBMSCs

The flow cytometry analysis detected the S-phase checkpoint between the HBMSCs and LPS treatment groups (1, 10, 100, 1000, and 10000 ng/ml LPS). No obvious differences were found (Figure 1A). The CCK-8 assay also demonstrated that various LPS concentrations had no effects on cell growth (Figure 1B). ALP and Alizarin Red staining showed that the osteogenic differentiation in HBMSCs was gradually inhibited by increasing LPS concentrations. Further, 100 ng/ml LPS markedly reduced the ALP level and matrix mineralization, and no further changes were found in the 10000 ng/ml group (Figure 1C). Based on these findings, the concentration of 100 ng/ml LPS was selected as the optimal level to mimic the inflammatory environment.

**Figure 1:** LPS had no effects on proliferation and inhibited osteogenic differentiation of HBMSCs (**A**) Flow cytometry analysis showed no effects of liposomes on the cell cycle of HBMSCs after 1, 3, and 5 days. (**B**) Cell viability assessed by CCK-8 showed that LPS did not affect cell proliferation. (**C**) Osteogenic differentiation assessed by ALP staining and Alizarin Red staining was inhibited under the stimulation of 100 ng/ml LPS, *n*=5.

### Effects of PTH on LPS-induced HBMSC proliferation

PTH (10^−7^, 10^−9^, 10^−11^, and 10^−13^ M) was added to HBMSCs with LPS treatment. No significant differences were found in cell viability and S-phase population among the control, LPS, and LPS + PTH groups (Figure 2A,B). Therefore, PTH had no effects on the proliferative ability of LPS-induced HBMSCs.

**Figure 2:** PTH had no effects on LPS-induced HBMSC proliferation (**A**) Cell viability of HBMSCs assessed by CCK-8 showed that PTH did not affect cell proliferation. (**B**) Flow cytometry analysis showed no effects of PTH on the cell cycle of HBMSCs after 1, 3, and 5 days, *n*=5.

### Screening for the optimal PTH concentration

After LPS treatment, HBMSCs were incubated with different concentrations of PTH (10^−7^, 10^−9^, 10^−11^, and 10^−13^ M). The 10^−9^ M PTH group showed the most elevated ALP amounts compared with other PTH groups, as confirmed by ALP activity and staining (Figure 3A,B). Meanwhile, Alizarin Red staining demonstrated that matrix mineralization was the highest in the 10^−9^ M PTH group, while other PTH groups showed no differences compared with the LPS group (Figure 3C). These results suggested 10^−9^ M as the optimal PTH level for evaluating osteogenic differentiation in LPS-induced HBMSCs.

**Figure 3:** A concentration of 10^−9^ M as the optimal PTH level on osteogenic differentiation in LPS-induced HBMSCs (**A**,**B**) ALP levels detected by ALP staining and activity assay showed that the concentration of PTH at which the osteogenic differentiation of HBMSCs was the strongest was 10^−9^ M. (**C**) Matrix mineralization determined by Alizarin Red staining also indicated that 10^−9^ M PTH was the best for osteogenic differentiation in LPS-induced HBMSCs. Data are mean ± SD. *P<0.05 and **P<0.01 versus the control (HBMSCs) group; ^##^*P*<0.01 versus the LPS (HBMSCs + LPS) group, *n*=5. Scale bar, 200 μm.

### Effects of PTH on LPS-induced osteogenic differentiation of HBMSCs

The effect of 10^−9^ M PTH on osteogenic differentiation in LPS-induced HBMSCs was further examined. ALP, COL1, OPN, OCN, and RUNX2 mRNA levels decreased on LPS administration, whereas PTH treatment resulted in opposite effects (Figure 4A). Meanwhile, Western blot analysis revealed that ALP, COL1, OPN, OCN, and RUNX2 protein levels were markedly lower in the LPS group than in the control group, while PTH reversed these inhibitory effects (Figure 4B). Besides, the expression of OCN and RUNX2 was obviously up-regulated in the PTH treatment group compared with the LPS group, as revealed by immunofluorescence (Figure 4C,D). Collectively, these results indicated that PTH enhanced the osteogenesis of LPS-induced HBMSCs.

**Figure 4:** PTH promoted osteogenesis in LPS-induced HBMSCs (**A**) Relative mRNA levels of ALP, COL1, OPN, OCN, and RUNX2 assessed by qRT-PCR suggested that PTH promoted osteogenesis-related gene expression. (**B**) Protein levels of ALP, COL1, OPN, OCN, and RUNX2, determined by Western blot analysis, also confirmed that the osteogenic ability of HBMSCs was elevated by PTH under the stimulation of LPS. (**C**,**D**) Expression levels of OCN and RUNX2 revealed by immunofluorescence were higher in the PTH (HBMSCs + LPS + PTH) group than in the LPS (HBMSCs + LPS) group. Data are mean ± SD. *P<0.05 and **P<0.01 versus the control (HBMSCs) group; ^#^*P*<0.05 and ^##^*P*<0.01 versus the LPS (HBMSCs + LPS) group, *n*=5. Scale bar, 50 μm.

### Role of the JNK MAPK pathway in PTH-induced osteogenesis

JNK, p-JNK, p38, p-p38, ERK1/2, and p-ERK1/2 protein levels were measured to investigate the role of MAPK signaling in PTH-associated processes. Compared with control untreated HBMSCs, LPS administration remarkably suppressed JNK phosphorylation. However, elevated p-JNK levels were detected in the PTH group compared with the LPS group, while p38, p-p38, ERK1/2, and p-ERK1/2 protein levels exhibited no distinct differences (Figure 5A). The ratio of p-JNK/JNK also indicated the activated JNK pathway after PTH treatment (Figure 5B). To further clarify the underlying mechanisms, SP600125, a specific inhibitor of JNK MAPK, was applied. SP600125 inhibited the beneficial effects of PTH in reversing JNK phosphorylation (Figure 5C). As expected, SP600125 reduced ALP activity and ALP-positive area driven by PTH (Figure 6A,B). Besides, Alizarin Red staining and qRT-PCR demonstrated that the mineralization and osteogenic gene expression levels droved by PTH were remarkably reduced on SP600125 administration (Figure 6B,C). In addition, the protein levels of osteogenic markers enhanced by PTH also decreased after SP600125 administration (Figure 6D–F). So far, the results demonstrated that PTH promoted the osteogenic differentiation of LPS-induced HBMSCs through the JNK MAPK pathway.

**Figure 5:** Impact of PTH on the MAPK pathway (**A**) p-JNK, JNK, p-p38, p38, p-ERK1/2, and ERK1/2 protein levels assessed by Western blot analysis. The expression of p-JNK was elevated in the PTH group compared with the LPS group, while p38, p-p38, ERK1/2, and p-ERK1/2 protein exhibited no distinct differences. (**B**) Relative phosphorylation level was measured by densitometry analysis using ImageJ software. (**C**) Protein amounts of p-JNK and JNK obtained by Western blot analysis on SP600125 treatment showed that PTH increased the expression of p-JNK. Data are mean ± SD. *P<0.05 versus the control (HBMSCs) group; ^#^*P*<0.05 versus the LPS (HBMSCs + LPS) group, *n*=5.

**Figure 6:** PTH promoted osteogenic differentiation by activating the JNK MAPK pathway (**A**,**B**) ALP levels detected by ALP staining and activity assay; mineralized matrix formation assessed by Alizarin Red staining. SP600125, a specific inhibitor of JNK MAPK, depleted the osteogenic ability of PTH under LPS stimulation. Scale bar, 200 μm. (**C**) Relative ALP, COL1, OPN, OCN, and RUNX2 mRNA amounts evaluated by qRT-PCR suggested that SP600125 reversed the promoting effects of PTH on osteogenesis-related gene expression. (**D**) Protein levels of ALP, COL1, OPN, OCN, and RUNX2, determined by Western blot analysis, indicated that the inhibition of JNK dampened the expression of osteogenesis-related proteins. (**E**,**F**) Expression levels of OCN and RUNX2 revealed by immunofluorescence were lower in the SP600125 (HBMSCs + LPS + PTH + SP600125) group than in the LPS (HBMSCs + LPS + SP600125) group. Scale bar, 50 μm. Data are mean ± SD. **P<0.01 versus the control (HBMSCs) group; ^#^*P*<0.05 versus the LPS (HBMSCs + LPS) group, *n*=5.

## Discussion

Alveolar bone regeneration plays a key role in treating periodontitis. The osteogenic differentiation property of mesenchymal stem cells in an inflammatory environment is important during this process. Accumulating evidence indicates that LPS serves as an inflammatory factor and impairs the formation of a localized osteogenic microenvironment by penetrating the periodontal tissue [26–28]. HBMSCs, which exhibit the advantages of extensive sources and low immunogenicity, are essential in alleviating bone complications [29]. Besides, HBMSCs also show considerable benefits in regenerating periodontal tissue according to their self-renewal and multiple differentiation properties [30]. Nevertheless, diminished osteogenesis, unexpected adipogenesis, and suppressed osteoblast-related gene expression have been reported in LPS-induced HBMSCs [31]. An inflammatory microenvironment formed by LPS was created to decrease the osteogenesis of HBMSCs in the present study, confirming previous findings [32]. Therefore, better strategies to reverse the inhibited osteogenic differentiation of HBMSCs might help design new approaches for treating periodontitis.

The influence of PTH on bone remodeling is well established [33]. PTH serves as an effective anabolic therapeutic in reducing the apoptosis and senescence of HBMSCs [34,35]. In addition, PTH also promotes HBMSC proliferation, maintains HBMSC integrity, and slows down age-related osteoporosis in adult mice by reversing HBMSC apoptosis [36]. Furthermore, daily injections of PTH result in a considerable increase in mass, strength, and mineral density of bone, contributing to the improvement in bone microarchitecture and healing of bone defect size [37]. We hypothesized that PTH could impede the pathophysiological processes in LPS-induced HBMSCs. First, we demonstrated that PTH did not affect the proliferative capacity of HBMSCs based on a series of experiments. Next, ALP staining and activity, qRT-PCR, and Western blot analysis indicated that 10^−9^ M PTH was optimal in reversing ALP inhibition caused by LPS, which represented an early osteogenic marker during mineralization [38]. COL1 represents an important structural protein displaying excellent osteoconductive function [39]. OPN is a regulator with a dual role in bone metabolism [40]. OCN is considered a late-stage osteogenic marker, reflecting the mature osteogenesis phenotype [41]. RUNX2 is a transcription factor that acts as an early-stage osteogenic marker in regulating bone tissue enrichment [42]. We further suggested that PTH rectified the inhibition of the aforementioned osteogenic markers by LPS. Based on Alizarin Red staining data, we concluded that PTH had a better effect in remolding LPS-induced HBMSCs.

The MAPK pathway was closely associated with PTH treatment. MAPK is a broad-based protein kinase that acts as an indispensable part of signal transduction [43]. Three major subfamilies of MAPK (ERK1/2, JNK, and p38) represent valuable triggers for the differentiation of mesenchymal stem cells [44]. As shown earlier, PTH elevated p-JNK levels in LPS-induced HBMSCs, highlighting the role of phosphorylated JNK in restoring bone deficiency. A specific pathway inhibitor was further applied, and the results confirmed that suppressing JNK MAPK significantly inhibited PTH-driven osteogenesis. Taken all these findings together, PTH promoted the osteogenic differentiation in HBMSCs against LPS through the JNK MAPK pathway.

In summary, these data uncovered a potential role for PTH in treating LPS-induced HBMSCs and provided novel insights into a potential strategy therapy of the inflammatory bone-destructive processes. Further *in vivo* experiments are needed to understand the detailed mechanisms better.

## Data Availability

The materials, data, and any associated protocols that support the findings of the present study are available from the corresponding authors upon request.

## Abbreviations

ALP: alkaline phosphatase
CCK-8: cell counting kit-8
COL1: collagen 1
DAPI: 4',6-diamidino-2-phenylindole
GAPDH: glyceraldehyde-3-phosphate dehydrogenase
HBMSC: human bone marrow mesenchymal stem cell
JNK: c-Jun N-terminal kinase
LPS: lipopolysaccharide
MAPK: mitogen-activated protein kinase
OCN: osteocalcin
OPN: osteopontin
PBS: phosphate-buffered saline
PTH: parathyroid hormone
RUNX2: runt-related transcription factor 2
